# The Effect of Intrinsic Mechanical Properties on Reducing the Friction-Induced Ripples of Hard-Filler-Modified HDPE

**DOI:** 10.3390/polym15020268

**Published:** 2023-01-04

**Authors:** Chuanbo Liu, Chengqing Yuan, Shutian Liu

**Affiliations:** 1 School of Mechanical and Electronic Engineering, Wuhan University of Technology, Wuhan 430070, China; 2 School of Transportation and Logistics Engineering, Wuhan University of Technology, Wuhan 430063, China; 3 Processing and Performance of Materials, Department of Mechanical Engineering, Eindhoven University of Technology, P.O. Box 513, 5600 MB Eindhoven, The Netherlands

**Keywords:** HDPE, Si_3_N_4_, ripple deformation, intrinsic mechanical property

## Abstract

Ripple deformations induced by friction on polymeric materials have negative effects on the entire stability of operating machineries. These deformations are formed as a response to contacting mechanics, caused by the intrinsic mechanical properties. High-density polyethylene (HDPE) with varying silicon nitride (Si_3_N_4_) contents is used to investigate different ripple deformation responses by conducting single-asperity scratch tests. The relationship between the intrinsic mechanical properties and the ripple deformations caused by filler modifications is analyzed in this paper. The results show the coupling of the inherent mechanical properties, and the stick-slip motion of HDPE creates ripple deformations during scratching. The addition of the Si_3_N_4_ filler changes the frictional response; the filler weakens the ripples and almost smoothens the scratch, particularly at 4 wt.%, but the continued increase in the Si_3_N_4_ content produces noticeable ripples and fluctuations. These notable differences can be attributed to the yield and post-yield responses; the high yield stress and strain-hardening at 4 wt.% provide good friction resistance and stress distribution, thus a smooth scratch is observed. In contrast, increasing the filler content weakens both the yield and post-yield responses, leading to deformation. The results herein reveal the mechanism behind the initial ripple deformation, thus providing fundamental insights into universally derived friction-induced ripples.

## 1. Introduction

Polymer-based materials are widely used in engineering because of their high resistance to fatigue, low weight, and low coefficient of friction (COF) making them a more suitable candidate than their metal counterparts for usage as frictional materials [1,2,3,4,5]. However, the capacity of polymers to guarantee high performance in long-term friction and wear patterns is constrained by intrinsic faults, such as low resistance to high temperatures and wear [6,7,8,9]. For example, friction-induced surface deformation leads to an unstable and unreliable frictional system, with large fluctuations in the frictional force and COF [10,11,12,13].

Therefore, numerous studies have been conducted to reduce or eliminate the number of friction-induced deformations on polymer surfaces. One effective method of reducing the number of friction-induced deformations is improving the lubricating conditions in areas where friction or wear occurs. For example, fillers with conventional two-dimensional structures, such as molybdenum disulfide, black phosphorus, and graphene, have been used to modify pure polymers and create lubricating films during friction [14,15,16,17,18]. Another reason behind polymer surface deformation is the unstable or uneven external force exerted during friction. To decrease the external force, multidimensional modification materials, such as tetra-needle-shaped ZnO and flower-like nanoparticles, are added to the polymer to increase its internal friction consumption [19,20,21,22].

Although functioned-filler modifications can lessen the deformation on the surfaces of polymer materials, insights into the formation mechanism behind surface deformations are still limited. Friction-induced deformation on the polymer surface represents the polymer’s inherent ability to resist the accumulation and release of local stress [23,24,25]. Deformation starts when the local stress begins to accumulate and exhibits an increasing trend, whereas stress release concludes the deformation cycle. These stress responses are governed by the intrinsic mechanical properties of the polymer, such as the yield stress, strain-softening, and strain-hardening [26,27]. Thus, understanding how polymer responses differ after modification can help reveal the formation mechanism of friction-induced deformations.

High-density polyethylene (HDPE), a frequently used engineering material with a simple molecular structure, is widely used as the pure matrix material for modification [28,29,30]. In addition, silicon nitride (Si_3_N_4_), a hard filler, is chosen as the modifying filler because of its proven self-lubricating property in specific frictional conditions [31,32,33]. Although the addition of Si_3_N_4_ has the ability to reduce the friction force and friction coefficient of the HDPE composites, the mechanism for the formation of the frictional-induced deformation is still lacking. In this case, the relationship between the addition of hard fillers, intrinsic mechanical properties (yield stress, strain-softening, and strain-hardening), and frictional responses (penetration depth, frictional force, and ripple deformation) is analyzed. The findings of this study can provide a vital link between the yield and post-yield responses of polymers and clarify the mechanism that causes surface deformation. These results will provide a framework on how to manage the friction-induced surface deformation of polymer-based composites, allowing for the synthesis of stable frictional systems.

## 2. Methods and Experiments

### 2.1. Experimental Materials and Sample Preparation

A high-density polyethylene (HDPE) blow-molding grade, with a melt flow index of 0.7 (190 °C/2.16 kg), is used as the matrix material in this study and was kindly provided by SABIC (B6246LS). The HDPE particles had an average diameter of 2 mm (Figure 1A). A silicon nitride (Si_3_N_4_) filler, with a diameter of 5 μm, was used to modify the internal structure of the HDPE, owing to its stable physicochemical properties (Figure 1B) [34]. All materials were provided by Aladdin Co., Ltd. (Shanghai, China). A double-screw extrusion granulation machine (ZC-65D, Nanjing Zhicheng Rubber Machinery Co., Ltd., Nanjing, China) was used to mix the HDPE and Si_3_N_4_ particles, and a uniform mixture was obtained (Figure 1C). The mixture was melted and compressed at 200 °C and 200 kN for at least 10 min in a hot-pressing molding machine, and two aluminum sheets were applied to guarantee the smooth surface of the HDPE sample (Figure 1D). The manufactured sample was put into ice water (0 °C) to ensure adequate cooling methods. The prepared samples were cut into the required size and shape for tensile (dumbbell shape with dimensions of 11.5 mm × 5 mm) and compression tests (cylinder shape with dimensions of 4 mm × 4 mm), as shown in Figure 1E,F. A single-asperity test was conducted by employing a scratching testing machine with a rigid diamond indenter (90°/50 μm) (Figure 1G). For the scratching sample, the mixture was melted on a hot stage at 200 °C for 10 min and manually compressed between two glasses to maintain a very low surface roughness. The pure HDPE sample has a mean surface roughness (Sa) of about 0.04 ± 0.01 m (White Light Interferometer, Micro Xam, ADEP Hase Shift, Inc., Tucson, AZ, USA). However, as the Si_3_N_4_ amounts are increased, this value exhibits an upward trend (from 0.041 ± 0.01 m in 2 wt.% to 0.052 ± 0.01 m in 8 wt.%).

Different Si_3_N_4_ contents (0, 2, 4, 6, and 8 wt.%) were added to the HDPE samples to investigate the relationship between the Si_3_N_4_ content and frictional responses of the HDPE composites.

### 2.2. Experimental Apparatus

The strain-stress responses were evaluated by conducting tensile and compression tests at three different strain rates of 0.001, 0.01, and 0.1 s^−1^. A load of 0.1 MPa was applied at the beginning of each tensile and compression test to ensure positive stress. The single-asperity scratch test was performed on a micro-indention tester to determine the frictional force and penetration depth. During the scratching test, the indenter tip remained in a stationary position at the top, whereas the HDPE composite was moved at various velocities from 0.1 to 100 mm/s. The applied normal load was 200 mN, and the sliding distance was 1 mm. Each test was repeated three times to ensure repeatability.

### 2.3. Measurement Techniques and Procedures

A micro indention tester (Micro Indenter, CSM Instruments SA, Peseux, Switzerland) was used to conduct the single-asperity sliding friction experiments, and an optical microscope (BX51-P, Olympus Corporation, Tokyo, Japan) was used to observe scratches after the sliding test. The scratch morphology was detected by using a confocal laser scanning microscope (Plμ2300, Sensofar Group, Barcelona, Spain) with a Nikon Plan Fluor 50 ×/0.80 EPI lens. The intrinsic mechanical properties, from both the tensile and compression tests, were determined by using a universal tensile tester equipped with a 10 kN load cell (Zwick Z010, ZwickRoell, Ulm, Germany). A ball-plate normal friction test was conducted by using a commercial tester (R-tec tribo-tester, Rtec Instruments Inc., San Jose, CA, USA). The micromorphology of the polymer scratch was investigated by using scanning electron microscopy (VEGA3, TESCAN, Brno, Czech Republic). Differential scanning calorimetry (DSC) measurements were also performed (DSC 823e, Mettler–Toledo. B. V., Tiel, The Netherlands).

## 3. Results and Discussions

### 3.1. Intrinsic Mechanical Properties of the HDPE Composites

The strain–stress responses of HDPE composites in the uniaxial tensile tests at different strain rates are displayed in Figure 2, and the yield stress and strain-stress curves are obtained. At a fixed strain rate of 0.1 s^−1^ (Figure 2A), the stress first shows an increasing trend until it reaches the yield point (yield stress) and then shows a noticeable drop called strain localization. The yield point and strain localization are highly dependent on the Si_3_N_4_ content of the HDPE composites. The yield stress first increases with the addition of Si_3_N_4_, reaching a peak value (26 MPa) at 4 wt.% Si_3_N_4_; however, a dramatic decrease occurs as more Si_3_N_4_ is added to the HDPE. Additionally, 8 wt.% Si_3_N_4_ causes the lowest yield stress of 21 MPa and shows a nonhomogeneous tensile stress after strain localization. Owing to the viscoelastic behavior of the polymer material [35,36], the strain-rate dependency generates a higher yield stress at high strain rates, and this phenomenon applies to all added contents of Si_3_N_4_ (Figure 2B). At less than 4 wt.% Si_3_N_4,_ increasing the yield stress strengthens the frictional resistance of the composite, allowing less indention depth. Notably, the addition of more Si_3_N_4_ beyond 4 wt.% decreases the frictional resistance of the composite.

A uniaxial compression test was conducted on the HDPE composite to obtain the true strain-stress response under different Si_3_N_4_ contents, and three parameters were observed (yield stress, strain-softening, and strain-hardening). Similar to the result from the tensile test, the yield stress exhibits an initial positive correlation with increasing Si_3_N_4_ content until a 4 wt.% content is reached. Once the additional Si_3_N_4_ content exceeds 4 wt.%, the yield stress lowers (Figure 3A). The viscoelastic behavior ensures that the yield stress increases with increasing strain rates; in the 4 wt.% Si_3_N_4_ composites, the yield stress increases from 41 MPa at 0.001 s^−1^ to 47 MPa at 0.1 s^−1^ (Figure 3B). Moreover, the addition of 4 wt.% Si_3_N_4_ contributes to the lowest value of strain-softening (Figure 3C), indicating that less stress is localized during contact, whereas higher strain-softening causes higher localization of stress and initiates deformation. However, strain-hardening may disperse the concentrated stress, stopping deformation. In the case of the composite with 4 wt.% Si_3_N_4_, the higher the strain-hardening, the more capable it is of distributing the limited stress, thus weakening the deformation (Figure 3D). However, when both high localization and low distribution of the contacting stresses are found together in a sample, significant deformation can be created.

### 3.2. Internal Structures of the HDPE Composites

The internal structures (lamella and crystalline) of semi-crystalline polymers, such as HDPE, are controlled by the melting and cooling processes after melting. During the cooling process, the crystalline phase tends to nucleate on impurities and additives and at the phase boundary, thus typically demonstrating slow growth. The DSC results confirm that the addition of Si_3_N_4_ has no influence on the melting temperature of the HDPE composites (Figure 4A). When the melt is cooled (Figure 4B), the crystallization temperature slightly increases from 121 °C to 124 °C because of the addition of fillers, indicating that the Si_3_N_4_ particle filler can function as a nucleating agent in the HDPE crystallization process. As a result, compared with the pure HDPE sample, the crystallization peak and area increase with the addition of 4 wt.% Si_3_N_4_, indicating that more crystals are generated. However, the addition of more filler reduces the crystallization phase by limiting the growth space of each crystallization. The different internal structures of the HDPE composites directly influence their intrinsic mechanical properties; for example, the yield stress is enhanced by the increase in crystallization, and the addition of Si_3_N_4_ weakens the crystallization network, thus decreasing the strain-hardening (Figure 2 and Figure 3).

### 3.3. Frictional Responses of the HDPE Composites

Single-asperity scratching tests were conducted on the HDPE composites with different amounts of Si_3_N_4_, and four different scratching velocities were set (0.1, 1, 10, and 100 mm/min). Figure 4A presents the complete curves of the penetration depth and the corresponding frictional force of the pure HDPE at a scratching velocity of 0.1 mm/min and a loading force of 200 mN. Under the effect of the applied normal load, the indenter tip first penetrates the HDPE material and forms the contact area at the initial stage of sliding. As the sliding process progresses, the indenter tip reaches the deepest depth and generates a larger contact area; thus, a greater amount of the material accumulates (bow wave). Owing to the viscoelastic nature of polymers, the accumulated material pushes the indenter tip upward, creating a stable area of contact until sliding is complete. As a result, the frictional force generated by the penetration depth shows corresponding behaviors because of the bow wave and then remains stable until the sliding process completes.

As previously discussed, the addition of Si_3_N_4_ (2 wt.% and 4 wt.%) strengthens the yield and post-yield responses; thus, a reduced indentation depth and a reduced contact area are created because the higher yield stress provides more frictional resistance. As a result, a lower penetration depth, along with its corresponding frictional force, is observed. This is best observed on the 4 wt.% Si_3_N_4_ composites at 13 μm and 128 mN during the stable period (Figure 5B,C) at 1 mm/min and 200 mN. However, the significantly decreased yield stress at higher contents of Si_3_N_4_ (6 wt.% and 8 wt.%) allows a deeper indentation depth; therefore, more contact areas cause an increase in material accumulation (forming a large bow wave) and local stress, generating a high penetration depth and friction force.

Figure 5D,E shows the strain-rate dependency, ensuring that the HDPE exhibits an increasing yield stress as the scratching velocity increases. Therefore, the HDPE composites experienced decreasing trends on both penetration depth and friction force. Additionally, the Si_3_N_4_ content of 4 wt.% provides the best yield response for each scratching velocity and the lowest penetration depth and friction force.

### 3.4. Ripple Deformation Response on the HDPE Frictional Surfaces

Periodical ripple deformation was observed during the stable sliding period of the HDPE composites, and this phenomenon was directly influenced by the addition of Si_3_N_4_. As depicted in Figure 6A,(A-1), the pure HDPE displays typical ripple deformation with height variations between −1 and 0.8 μm, showing a decreasing trend with the addition of Si_3_N_4_, and the best performance occurs in the 4 wt.% Si_3_N_4_ composite, with ranges from −0.3 to 0.2 μm (Figure 6C,(C-1)). However, the addition of more Si_3_N_4_ beyond 4 wt.% shows a negative correlation, thus causing a more notable and fluctuating ripple deformation and increasing the ripple height to more than 2 μm (6 wt.% and 8 wt.%). This means that more materials are accumulated for higher ripple deformation, but the frequency of ripple deformation is reduced to a certain extent (Figure 6D–(E-1)).

The ripple deformation represents the accumulation and distribution of the sliding stress, and the stick-slip motion is periodic in nature. The intrinsic mechanical properties of HDPE, such as its yield and post-yield responses, determine the resistance of the polymer to deformation, thus influencing the ripple deformation response. After the yield point is reached, a process known as strain-softening allows stress to localize, thus generating the initial deformation; any subsequent increase in stress (strain-hardening) distributes the localized stress and completes the deformation (Figure 3). In this case, the low strain-softening and high strain-hardening exhibited by the 4 wt.% Si_3_N_4_ composite ensure that the low accumulated stress can be distributed more evenly, leading to the generation of a ripple deformation with a low height (H) and length (L) (Figure 7). In contrast, increased strain-softening and low strain-hardening with higher contents of Si_3_N_4_ (6 wt.% and 8 wt.%) result in more localized stresses that cannot be dispersed. As a result, more strains create a greater accumulation of material and noticeable ripples.

### 3.5. Influence of the Micro Ripple Responses from the Scratch Test to the Universal Friction Test

A single-asperity sliding test was performed to simulate the micro-frictional condition of the HDPE composites under various Si_3_N_4_ contents. A periodic ripple deformation was observed. In this case, a universal ball-plate friction test was conducted on the modified HDPE composite to verify the connection between the micro- and macro-frictional responses. During the universal ball-plate friction test, a stainless-steel ball with a radius of 10 mm was kept stable, while the HDPE composites were moved with a rotation driver below (Figure 8(A-4)). The frictional conditions were as follows: a velocity of 0.021 m/s, an applied normal load of 80 N, and a duration of 1800 s. After the ball-plate friction test, conventional and periodic ripple deformations with averaged 4.2 μm on ripple height were observed on the pure HDPE frictional surface (Figure 8(A-3)). As previously noted, the height variation of the ripples resulted from a direct correlation between the variation in frictional force and the created COF, which has an amplitude of △A (0.14) (△A is defined as the amplitude of the COF which explained in Figure 8(C-4)) (Figure 8(A-4)). Similar to the ripple responses from the single-asperity test on pure HDPE, the addition of Si_3_N_4_ reduced the ripple deformation on the frictional surface after ball-plate friction. The addition of 4 wt.% Si_3_N_4_ decreased the amplitude of the ripple (2.1 μm in Figure 8(B-3)), smoothed the frictional surface (Figure 8(B-2)), and stabilized the COF at low amplitudes (△A at 0.09 in Figure 8(B-4)). Higher Si_3_N_4_ contents, however, showed considerably inferior intrinsic mechanical properties, which led to noticeable and fluctuating ripples with large diameters after single-asperity sliding (Figure 8C,(C-1)). Although the frequency of these deformations occurring was low, these deformations produced more noticeable ripples on the friction surface (Figure 8(C-2,C-3)) and significantly raised the COF with fluctuations of approximately 0.3 (△A) (Figure 8(C-4)). Repeated contact mechanics aggravated the single-asperity-test-based ripple deformation because the universal friction test was complicated, and the increased ripple height and length fluctuated the COF response; however, the ripple frequency was not influenced [37,38]. However, the connection between a universal friction scenario and the conditions examined in this study was not investigated.

### 3.6. Influence of the Intrinsic Mechanical Properties on Ripple Deformation

The relationship between the intrinsic mechanical properties and the formation of ripples on the HDPE sliding surface is illustrated in Figure 9. At the start of the sliding test, the indenter tip first penetrates the HDPE surface and forms a contact area with the polymer (Figure 9A); this behavior is governed by the yield stress. The high frictional resistance generated by the high yield stress prevents the indenter from penetrating further into the polymer surface, thus reducing the contact area. As the scratching velocity is applied, a stress-increasing zone is formed at the front of the indenter tip, causing mutual movement between the indenter tip and the polymer. This behavior ends after the increasing stress exceeds the critical stress from the polymer itself, resulting in the commencement of the moving field. In this field, a complex situation arises because the materials begin to accumulate in front of the indenter tip, initiating ripple formation. This phenomenon can be attributed to the compression effect [39] (Figure 9B). The balance between strain-softening and strain-hardening determines the accumulation of materials. High strain-softening allows for more stress localization, which creates more strains on the contacting area, and therefore, more materials accumulate. Strain-hardening strengthens the material’s resistance by facilitating stress distribution and halting the ripple deformation process (the maximum ripple height, Hm, is generated), as shown in Figure 9B). The accumulated material experiences a tensile effect after the indenter tip slips over it, and a tensile effect zone is created (Figure 9C). The accumulated material begins to move as the applied tensile stress exceeds its maximum tensile yield stress; thus, the homogenous tensile deformation decreases the height and increases the length of the accumulated materials. Consequently, the observed ripple size height (H) and length (L) stop increasing.

This result reveals that the intrinsic mechanical properties, influenced by the addition of Si_3_N_4_, determine the ripple responses on the HDPE surface. The addition of 4 wt.% Si_3_N_4_ contributes to a higher yield stress to prevent deeper penetration into the HDPE surface; thus, a smaller contact area produces less stress during sliding. Moreover, the subsequent low strain-softening and high strain-hardening ensure that the localized stress can be better distributed, resulting in low material accumulation and less ripple deformation (Figure 3, Figure 6 and Figure 8). In contrast, the low yield and post-yield responses exhibited in the samples with higher Si_3_N_4_ contents (6 wt.% and 8 wt.%) lead to more localized stress on the contacting area, causing a higher accumulation of materials. Consequently, large ripple deformations are created, which fluctuate the COF (Figure 8 and Figure 9D,E).

## 4. Conclusions

In this study, the relationship between intrinsic mechanical properties and ripple deformation in HDPE composites with varying Si_3_N_4_ contents was investigated. The friction-induced ripple deformation during the sliding process indicated the periodic accumulation and release of the local stress, which was influenced by the responses of the yield and post-yield (the balance of strain-softening and strain-hardening). With the addition of Si_3_N_4_ (2 wt.% and 4 wt.%), a lower penetration depth and frictional force were observed because the increasing yield stress contributed to a higher frictional resistance. Furthermore, low strain-softening and high strain-hardening prevented strain localization and provided better stress distribution. This resulted in fewer materials being deformed, leading to smooth scratches with low ripples being observed (at 4 wt.%). However, higher Si_3_N_4_ contents (6 wt.% and 8 wt.%) in the HDPE affected the internal structure and forming process, resulting in weakened intrinsic mechanical properties. Owing to the low frictional resistance caused by the lower yield stress, deeper penetration occurred. In addition, the presence of a high localized strain (high strain-softening) and low distributed stress (low strain-hardening) caused a greater accumulation of stresses at the front of the indenter tip during the sliding process, leading to the formation of the HDPE composites and the occurrence of noticeable and fluctuating ripples.

## Figures and Tables

**Figure 1:** Sample preparation and testing apparatus: (**A**) HDPE granules; (**B**) silicon nitride powder (Si_3_N_4_); (**C**) double-screw extrusion granulation for mixed particles; (**D**) hot-pressing molding machine for testing the samples. Tensile (**E**) and compression (**F**) tests for the intrinsic mechanical property. (**G**) Frictional response from the single-asperity scratching test.

**Figure 2:** Strain-stress responses (from the tensile test) of the HDPE composites with different Si_3_N_4_ contents: (**A**) strain-stress curves and (**B**) yield stresses with different strain rates.

**Figure 3:** True strain-stress from the compression test of the HDPE composite: (**A**) complete strain-stress curve; (**B**) true yield stress, (**C**) strain-softening, and (**D**) strain-hardening, under different Si_3_N_4_ contents and strain rates.

**Figure 4:** DSC results of the HDPE composites with a rate of 10 ℃/min: (**A**) melting curves and (**B**) cooling (crystallization) curves.

**Figure 5:** Frictional responses of the HDPE composites with different Si_3_N_4_ contents: (**A**) penetration depth and corresponding frictional force; (**B**) penetration depth and (**C**) frictional force with increasing applied loads; (**D**) averaged frictional force and (**E**) penetration depth under different scratching velocities.

**Figure 6:** The ripple deformation response of the HDPE composites with different Si_3_N_4_ contents: (**A**,**A-1**) are 0 wt.%; (**B**,**B-1**) are 2 wt.%; (**C**,**C-1**) are 4 wt.%; (**D**,**D-1**) are 6 wt.%; (**E**,**E-1**) are 8 wt.%.

**Figure 7:** Ripple size: (**A**) height H and (**B**) length L of the HDPE composites with different Si_3_N_4_ contents.

**Figure 8:** Frictional responses of the HDPE with different contents of Si_3_N_4_ from the single-asperity test and the universal friction test: (**A**–**A-4**) 0 wt.%; (**B**–**B-4**) 4 wt.%; (**C**–**C-4**) 8 wt.%.

**Figure 9:** (**A**–**C**) graphically represent ripple deformation during the single-asperity scratch test; (**D**,**E**) show the relationships between the addition of Si_3_N_4_ and the intrinsic mechanical properties, the ripple, and COF responses.

## Data Availability

The data presented in this study are available on request from the corresponding author.
